# Skeleton-Based Action Recognition Based on Distance Vector and Multihigh View Adaptive Networks

**DOI:** 10.1155/2021/1507770

**Published:** 2021-08-18

**Authors:** Min Zhang, Haijie Yang, Pengfei Li, Ming Jiang

**Affiliations:** School of Computer Science, Hangzhou Dianzi University, Hangzhou 310000, China

## Abstract

Skeleton-based human action recognition has attracted much attention in the field of computer vision. Most of the previous studies are based on fixed skeleton graphs so that only the local physical dependencies among joints can be captured, resulting in the omission of implicit joint correlations. In addition, under different views, the content of the same action is very different. In some views, keypoints will be blocked, which will cause recognition errors. In this paper, an action recognition method based on distance vector and multihigh view adaptive network (DV-MHNet) is proposed to address this challenging task. Among the mentioned techniques, the multihigh (MH) view adaptive networks are constructed to automatically determine the best observation view at different heights, obtain complete keypoints information of the current frame image, and enhance the robustness and generalization of the model to recognize actions at different heights. Then, the distance vector (DV) mechanism is introduced on this basis to establish the relative distance and relative orientation between different keypoints in the same frame and the same keypoints in different frame to obtain the global potential relationship of each keypoint, and finally by constructing the spatial temporal graph convolutional network to take into account the information in space and time, the characteristics of the action are learned. This paper has done the ablation study with traditional spatial temporal graph convolutional networks and with or without multihigh view adaptive networks, which reasonably proves the effectiveness of the model. The model is evaluated on two widely used action recognition benchmarks (NTU-RGB + D and PKU-MMD). Our method achieves better performance on both datasets.

## 1. Introduction

Human action recognition is currently one of the most important tasks in computer vision, and it is widely used in human-computer interaction, video surveillance, video understanding [1], and virtual reality [2–4]. According to the different types of data input to the network [5], human action recognition can be roughly divided into two research directions. One is the RGB-based method, which has been widely used. The other is based on the 3D skeleton method; that is, the human body is represented by joints in 3D space, which has attracted more and more attention. Past studies have shown that using 3D skeleton data to represent human movements is very effective and robust and also is conducive to computer storage and calculation [6, 7], and the skeleton data are usually obtained by the video-based pose estimation method [8].

Most of the previous methods encode the position of the joints in each frame of the video, convert them into feature vectors, and perform pattern learning [9–12]. However, these methods ignore the potential connections between joints and thus lose a lot of movement information. In order to solve this problem, a method for constructing a skeleton graph is proposed to capture the dependencies between joints, in which each joint is used as a vertex of the graph, the connection between two joints is used as an edge, and the graph convolutional network (GCN) is used to extract the features [13]. However, the method does not take the spatial and temporal information into consideration, so ST-GCN [14] is proposed to learn both spatial and temporal information. The network divides the joints into several parts to use different convolution kernels for convolution. Although this method distinguishes the joints in different regions, it does not subdivide the relationship between the current joint and every other joints which will cause wrong recognition of some special actions. In real scenes, the height of video shooting is often different. For example, the angle of the video monitored by the camera is from top to bottom. Because of their different heights, the content presented by the same action is in variation, so training the actions data only at a single height is often not very robust.

In order to solve the above problems, this paper proposes a human action recognition method based on distance vector and multihigh view adaptive networks. First, the best observation view at different heights is automatically determined through the multihigh view adaptive networks, and the keypoints coordinates under the new observation view are formed. Then, the distance vector is calculated between each keypoint in the same frame and other keypoints and the distance vector between the same keypoints in different frames, where the distance vector includes the relative spatial distance and the relative spatial orientation. Next, spatial temporal graph convolutional networks are constructed that use joints as graph nodes and the connections between joints as edges, and finally the corresponding action category is obtained through the standard SoftMax classifier. The resulting network is illustrated in Figure 1.

The advantages of the network in this paper compared with other current networks are as follows. (1) The distance vector mechanism is introduced on the basis of the spatial temporal convolutional network, which can not only learn the information of the action in time and space but also obtain the correlation information between the keypoint and all other keypoints and realize the global association. (2) Multihigh adaptive networks are constructed to learn the keypoints information of the best observation view at different heights, under the premise of ensuring that the network is easier to learn features, and the generalization of the model is increased and the accuracy is improved. (3) The final model performs well on two popular datasets (NTU-RGB + D and PKU-MMD) and demonstrates the effectiveness of DV-MHNet.

## 2. Related Work

Recently, graph-based models have attracted more and more attention because of their ability to effectively represent graph data structures [15]. The current graph models mainly fall into two architectures: one framework named graph neural network (GNN), which is composed of graphs and recurrent neural networks. It is learned through multiple iterations of message passing and node states updating. It can capture the semantic relation and structural information within its neighbor nodes. In [16], the interaction between people and objects in video images is understood by using graph neural networks. In [17], GNN is used to establish dependencies between roles and predict a consistent structured output for situation recognition. The other is the graph convolutional network (GCN), which applies neural networks to the graph. Among them, the GCNs are divided into spectral GCNs and spatial GCNs. Spectral GCNs transform graph signals on graph spectral domains and then apply spectral filters on spectral domains. In [13], a semisupervised classification based on GCN is proposed, which determines the convolutional network structure through the local first-order approximation of spectral graph convolutions. For spatial graph convolution, the convolution operation is performed through the domain information of each node to obtain the new feature vector of each node. Martin and Nikos [18] formulated a convolution-like operation on graph structure. It is a weighted average operation with the conventional two-dimensional image convolution operation. In addition to extracting spatial information, video-based action recognition must also extract temporal information. In order to capture the spatial temporal characteristics of the graph sequence, the article [19] introduces for the first time a graph convolution LSTM with a cyclic structure, which is an extension of graph convolution.

Because skeleton data are robust to illumination change and scene variation, human action recognition methods based on skeleton data have received increasing attention. These approaches can be categorized into handcrafted feature-based methods and deep learning methods. For the first method, the authors in [20] used the relative 3D rotation between each body part to represent each joint, and the authors in [12] used the relative 3D geometry between all pairs of body parts to represent the human body skeleton. For human action recognition based on deep learning, Du et al. [9] divided it into five parts according to the physical structure of the human body and then input them into the hierarchical recurrent neural network for action recognition. Reference [21] introduced a view adaptive model suitable for skeleton sequences, which can adjust the observation perspective itself to a suitable perspective. In the work of [6, 22, 23], it can be found that for human action recognition tasks, it is not only necessary to obtain the spatial features of the skeleton but also the temporal features, which are equally important. Based on the above work, Yan et al. [14] formulated a human action recognition method based on spatial temporal graph convolution, which can automatically learn spatial and temporal features from the data, which makes the model have strong expression and generalization capabilities. In addition, human action recognition based on local graph convolutional network [23] learns by dividing the skeleton into several parts, which better captures the structural information of the skeleton. Different from [14] and [23], [22] captures the spatial structure information by the GCN while using LSTM to model the skeleton temporal details. Although the above methods have significantly improved the performance of human action recognition, they ignore the potential relations between different joints in the same frame and the same joint in different frames, and they do not enhance the skeleton image from multiple views which result in the lower recognition accuracy.

## 3. Method

This paper proposes a human action recognition method based on distance vector and multihigh view adaptive network, which mainly includes three parts: multihigh view adaptive network, distance vector calculation, and spatial temporal graph convolutional network. This section first introduces the construction of multihigh view adaptive network, then explains the calculation of distance vector, and finally introduces the construction of spatial temporal graph convolutional network.

### 3.1. Multihigh View Adaptive Network

The joint content under different views is very different. For the same action, due to the change of the angle, the recognition difference is caused. For example, in the field of surveillance video, the joint information at a high view is also very different from the joint information at a horizontal view. In order to eliminate the influence caused by the difference in perspective, a variable view network architecture is constructed to automatically reobserve the skeleton from a new virtual perspective before performing action recognition. Inspired by [24], the new joints coordinates are obtained by rotating the view, but it is just to find a better perspective for the data to generate new joints coordinates and then send it to the network for classification. In this article, the coordinates of the keypoints generated under the best views of different heights are sent to the network for training, and the height is expressed by the angle with the horizontal.  Figure 2 shows the best views at different heights. It can be seen that this is a bending action sequence. The first row is four frames of images extracted from the original video. The second row is the original keypoints and the corresponding human body motion modeling. The third row is the best view when the angle between the viewing angle and the horizontal is 0°. It can be found that the converted skeleton information is easier to learn, but the action has not changed. The fourth and fifth rows are the best views when the angle of view and the horizontal angle are *θ*_1_ and *θ*_2_, respectively, *θ*_2_ > *θ*_1_. It can be found that the best viewing angles at different heights are also different. By transforming the keypoints, the keypoints at different height views are obtained, and they are trained together to achieve the purpose of data enhancement.

Given the skeleton sequence *S* in the three-dimensional coordinate system, the *i*_*th*_ joint of the *k*_*th*_ frame is expressed as *v*_*k*,*i*_=[*x*_*k*,*i*_, *y*_*k*,*i*_, *z*_*k*,*i*_]^*T*^,  *k* ∈ (1,…, *K*), *i* ∈ (1,…, *N*). *K* refers to the total number of frames in a bone sequence, and *N* refers to the total number of joints in a frame. Because the coordinates of the joints in different frames will change, in the new coordinate system, the coordinate of the keypoint is *v*_*k*,*i*_ − *d*_*k*_, where *d*_*k*_ is the displacement of coordinate system. A new observation view is obtained by rotating counterclockwise around the*X* − *axis*, *Y* − axis, and *Z-*axis; the rotation angle is  *R*_*k*,*θ*_=[*α*_*k*,*θ*_, *β*_*k*,*θ*_, *γ*_*k*,*θ*_]; all joints in the same frame share the rotation angle, so the coordinates of the joints under the new view are expressed as follows:

(1) $$\begin{array}{c} v_{k,i,\theta }^{\prime }={\left[x_{k,i,\theta }^{\prime },y_{k,i,\theta }^{\prime },z_{k,i,\theta }^{\prime }\right]}^{T}=R_{k,\theta }\left(v_{k,i}-d_{k}\right). \end{array}$$

By constructing the multihigh perspective adaptive network to automatically learn and determine the best observation views at different heights, a series of keypoints positions under new perspectives can be obtained, which can be expressed as follows:

(2) $$\begin{array}{c} V=\left\{v_{k,i,\theta }^{\prime }|\theta \in \left\{0^{\circ },\theta_{1},\theta_{2},\ldots \right\}\right\}, \end{array}$$

where *θ* is the horizontal angle between different heights and the best view. According to the actual situation of the surveillance video, set the angle reasonably and use the DVST-GCN to recognize the skeleton information features generated by the MHNet. The MHNet is mainly composed of two LSTM network branches and a fully connected layer, one of which learns the rotation matrix of the joint where rotation matrix is *R*_*k*,*θ*_ and the another branch learns the displacement of joints at different heights, that is, under different *θ*, the learned *d*_*k*_. Finally, the three-dimensional coordinates of the joints under the new perspective are calculated by formula (1), and the schematic diagram and architecture diagram of the MHNet are shown in Figures 3 and 4.

As shown in Figure 4, the original skeleton coordinates of a certain frame of the video are input to the network and the main network is mainly composed of two LSTM branch networks. The first LSTM network is used to determine the displacement **d**_**k**_ under the specified angle, and the other LSTM network is used to learn and determine the appropriate perspective, that is, to obtain the rotation parameters *α*_**k**,*θ*_, *β*_**k**,*θ*_,  and *γ*_**k**,*θ*_. Among them, the three parameters are, respectively, expressed as the angle of rotation around the **x**, **y**, and **z** axes. After the rotation parameters and the displacement at the specified angle are obtained, the skeleton coordinate data are rotated and transformed according to the parameters to obtain a new skeleton coordinates. Then, the new set of skeleton coordinate points and the corresponding action labels are input into a network composed of multiple LSTMs, the skeleton data are learned from end to end, and after the features are fully connected, the output is finally obtained through the SoftMax function.

### 3.2. Skeleton Graph Structure

The human body is in motion for a period of time through the human pose estimation method to get the joints in each frame.  Figure 5 shows the skeleton graph information of several frames. We construct a spatial temporal graph **G**=(**V**, **E**) on a skeleton sequence with **N** joints and **K** frames, and its node set is **V**={**v**_**ki**_*| ***k**=1,…, **K**, **i**=1,…, **N**}. The black dot in Figure 5 represents the **i**_**th**_ joint in the **k**_**th**_ frame. According to the human body structure, the joints of each frame are connected to form a spatial edge **Es**={**v**_**ki**_**v**_**kj**_*|*(**i**, **j**) ∈ **B**}, where **B** is the set of all joints in the **k**_**th**_ frame, as shown in the red edge of Figure 5. The same nodes are connected in two consecutive frames into edges to form temporal edges **Et**={**v**_**ki**_**v**_(**k**+1)**i**_}, the green side as shown in Figure 5.

### 3.3. Spatial Temporal Graph Convolutional Network-Based Distance Vector

The input feature vector of the spatial temporal graph convolutional network is generally composed of the coordinate vector of the node and the estimated confidence. For the spatial temporal graph convolutional network based on the distance vector, it is necessary to consider the changes in the spatial distance and direction of all the keypoints in the same frame and all the same keypoints in different frames and describe a series of changes in the action more explicitly. The distance vector proposed in this paper is mainly composed of the distance between the keypoints and the relative direction of the keypoints. The distance between the keypoints can be expressed as follows:

(3) $$\begin{array}{c} L\left(v_{mi},v_{mj}\right)=\sqrt{{\left(x_{mi}-x_{mj}\right)}^{2}+{\left(y_{mi}-y_{mj}\right)}^{2}+{\left(z_{mi}-z_{mj}\right)}^{2}},\;i,j\in \left(1,\ldots ,N\right), \end{array}$$

(4) $$\begin{array}{c} L\left(v_{mi},v_{ni}\right)=\sqrt{{\left(x_{mi}-x_{ni}\right)}^{2}+{\left(y_{mi}-y_{ni}\right)}^{2}+{\left(z_{mi}-z_{ni}\right)}^{2\;}},\;i,j\in \left(1,\ldots ,N\right), \end{array}$$

where (*x*, *y*, *z*) is the coordinate of the keypoint, and formula (3) represents the spatial distance between the *i*_th_ keypoint and the *j*_th_ keypoint in the same frame, and formula (4) represents the spatial distance between *i*_th_ keypoints of *m*_th_ frame and the *i*_th_ keypoint of the *n*_th_ frame. The relative position between the keypoints can be expressed as follows:

(5) $$\begin{array}{c} \overset{⟶}{r}\left(v_{mi},v_{mj}\right)=\left(\left(x_{mi}-x_{mj}\right),\left(y_{mi}-y_{mj}\right),\left(z_{mi}-z_{mj}\right)\right),\;i,j\in \left(1,\ldots ,N\right), \end{array}$$

(6) $$\begin{array}{c} \overset{⟶}{r}\left(v_{mi},v_{ni}\right)=\left(\left(x_{mi}-x_{ni}\right),\left(y_{mi}-y_{ni}\right),\left(z_{mi}-z_{ni}\right)\right),\;i,j\in \left(1,\ldots ,N\right), \end{array}$$

where (*x*, *y*, *z*) is the coordinate of the keypoint and $\overset{⟶}{r}$ is a direction vector. Formula (5) represents the position of the *j*_th_ keypoint relative to the *i*_th_ keypoint in the same frame, and formula (6) represents the orientation of the *i*_th_ keypoint in the *n*_th_ frame relative to the *i*_th_ keypoint in the *m*_th_ frame. As shown in Figure 6, assuming figure (a) is the *n*_th_ frame image of the video and figure (b) is the *n*+1_th_ frame image of the video, for the *K*_1_ skeleton point of the *n*_th_ frame, the distance vector between it and other keypoints is represented by the dotted line. The arrows indicate that the dashed arrows from *K*_1_ to *K*_2_ indicate the distance vectors between the same keypoints in different frames. It can be seen from the figure that in the *n*+1_th_ frame, the distance between the keypoint *K*_2_ and the keypoint *F*_2_ is closer, and the direction is slightly changed. By constructing the distance vectors between keypoints, the change information of the action can be effectively captured, and learning can be carried out through the spatial temporal graph convolutional network.

Therefore, the distance vector between keypoints, the coordinate position of the joint, and the confidence of the joint form a new input feature vector *F*_new_(*v*_*ti*_). Taking the common two-dimensional image convolution operation as a reference, the spatial temporal graph convolution operation can be written as follows:

(7) $$\begin{array}{c} F_{\text{out}}\left(v_{mi}\right)=\sum_{v_{mj}\in B\left(v_{mi}\right)}\frac{1}{Z_{mi}\left(v_{mj}\right)}F_{\text{new}}\left(p\left(v_{mi},v_{mj}\right)\right)\cdot w\left(v_{mi},v_{mj}\right),\\ F_{\text{out}}\left(v_{mi}\right)=\sum_{v_{ni}\in B\left(v_{mi}\right)}\frac{1}{Z_{mi}\left(v_{ni}\right)}F_{\text{new}}\left(p\left(v_{mi},v_{ni}\right)\right)\cdot w\left(v_{mi},v_{ni}\right), \end{array}$$

where *B*(*v*_*mi*_) is the domain constraint condition of the joint. For spatial graph convolution, *B*(*v*_*mi*_)={*v*_*mj*_*|d*(*v*_*mj*_, *v*_*mi*_) ≤ *D*}, *d*(*v*_*mj*_, *v*_*mi*_) represents the shortest distance from *v*_*mj*_ to *v*_*mi*_. For temporal graph convolution, *B*(*v*_*mi*_)={*v*_*ni*_*|d*(*v*_*ni*_, *v*_*mi*_) ≤ *K*, |*n* − *m*| ≤ Γ/2}, where *K*is the size of the convolution kernel and Γcontrols the size of the convolution kernel in the temporal domain. *p*  is the sampling function to obtain the neighbor joint centered on the joint, *w*  is the weight function, and *Z*  is the normalization item.

## 4. Experiment

*Datasets*. We evaluated our proposed method on two popular datasets (PKU-MMD and NTU-RGB + D). Among them, the PKU-MMD datasets contain more than 1,000 video clips, a total of 52 action categories, and 66 objects are completed in three camera views. The NTU-RGB + D datasets contain 56,000 video clips, covering more than 60 actions and filmed by 40 volunteers in a limited laboratory environment. The datasets provide the 3D joint positions (**x**, **y**, **z**) in the camera coordinate system.

*Experimental Settings*. For better experiments, the joints are rotated by a certain angle around *x*, *y*, and *z*. These angles are randomly generated between −90 and 90°. In addition, in order to simplify the experiment, we removed unnecessary keypoints. The initial learning rate of the two datasets is set to 0.005. In order to alleviate the overfitting problem, the probability of dropout is set to 0.5, the initialization parameter of the fully connected layer is set to 0, and the Adam optimizer is used to train the networks.

*Evaluation Criteria*. For the NTU-RGB + D datasets, the author of the datasets recommends two benchmarks: one of them is *X*-Sub, which includes 39889 training sets and 16390 verification sets. The training sets come from an actor's clip and the evaluation sets clips from other performers. The other is *X*-View, which includes 37462 training sets and 18817 validation sets. The training sets come from the second and third views of the camera and the validation sets come from the first view of the camera. For PKU-MMD datasets, there are also two recommended evaluate protocols, i.e., X-Sub and X-view. For detection-specific hyperparameters, we basically follow the settings in [25]. In particular, we use anchor scales of {50, 100, 200, 400} in the temporal proposal network.

## 5. Results

### 5.1. Evaluation

*Results on the NTU-RGB* *+* *D Datasets*.  Table 1 presents the results on the NTU-RGB + D datasets X-Sub and X-view. We have compared MH-DVNet with some advanced methods. In particular, our method is better than a series of spatial temporal graph convolutional networks, with an accuracy of 95.3% in X-Sub and 89.5% in X-view. In addition, it can be seen from the table that the accuracy of the VA-LSTM [21] method and ST-GCN [14] method is lower than that of the model proposed in this paper, which proves that this model is indeed improved on their basis.

*Results on the PKU-MMD Datasets*. There are few papers using this dataset, but the model has achieved good results.  Table 2 shows the accuracy of the MH-DVNet on the PKU-MMD datasets. The model achieves relatively good performance with an accuracy of 92.7% in X-Sub and 94.4% in X-view.

### 5.2. Ablation Study

We take the ST-GCN [14] as the benchmark model and conduct an ablation study on the X-Sub and X-View verification sets of NTU-RGB + D.

*DVNet*. We evaluated the following two models together: ST-GCN (benchmark model) and DVNet; the latter is improved based on ST-GCN. The benchmark model does not use the distance vector between each keypoint and other keypoints but defines a division method to classify several joints into one category. By calculating the distance vector between each keypoint of the current frame and the distance vector of the same keypoint in different frames, the change information of the action can be effectively captured. We did a comparative test on the NTU-RGB + D verification sets, as shown in Figure 7, and we can find that our proposed method is better than the ST-GCN.

*MHNet*. In the same way, we conducted a comparative experiment on the two cases where the MHNet generates joint coordinates in multiple views and directly uses the joint coordinates in a single view. Through the MHNet, it can generate the best view of different heights, which not only ensures that the best action characteristics can be learned but also can ensure recognition accuracy under high viewing angles such as some monitoring fields.

According to the actual scene, we reasonably increased the angle of view with 10° steps each time to train the model in stages. The final model and ST-GCN and VANet were ablated experiments. The experimental results are shown in Figure 8, and it can be found that the MHNet has the best effect.

In addition, since DVNet and MHNet have achieved better results under the benchmark model, we have reason to merge the two into the benchmark model and conduct a comparative test on the NTU-RGB + D verification set. As shown in Figure 8, it can be found that this method is better than the benchmark model.

## 6. Conclusion

In this paper, an action recognition method based on MH-DVNet is proposed, which mainly succeeds in the following three aspects. (1) The MHNet is used to automatically determine the best observation of different heights and generate multiple joints coordinates combinations under the same action category, which improves the accuracy while also improving the specific scene robustness. (2) Using the distance vector between each keypoint to capture the change information of the action, it can learn a wealth of linkage features and improve the accuracy on the basis of the ST-GCN. (3) We have done a lot of ablation experiments and reasonably proved the effectiveness of MH-DVNet.

## 7. Further Study

The method proposed in this paper has good robustness to the action information from different perspectives, so the complexity of the model is relatively large. In the future, we will try to reduce the complexity of the model without reducing the accuracy. In addition, this model can further improve the accuracy; a one-hot encoding technique [35] is used to convert the categorical data values to binary form. This is followed by the implementation of a crow search algorithm (CSA) for selecting optimal hyperparameters for training of dataset using the convolution neural networks. This method can be used to transform the action classification information into binary information and train a better model. Furthermore, a novel multidirectional long short-term memory (MLSTM) technique [36] is being proposed to predict the stability of the smart grid network. It has higher accuracy than the traditional LSTM, so it can be used to determine the best view of action, so as to improve the accuracy.

## Figures and Tables

**Figure 1:** The network architecture diagram proposed in this article including multihigh adaptive networks, calculated distance vector, and spatial temporal graph networks.

**Figure 2:** The best keypoint representation under the same action at different height angles.

**Figure 3:** MHNet schematic diagram. (a–c) New perspectives at different heights. Among them, (a) is the best view determined by the adaptive network, and (b) and (c) are the best view under the condition of adding angle constraints. From frame 1 to frame *t* the posture of the human body is constantly changing, and the MHNet can always find the best view for learning.

**Figure 4:** This figure is the MHNet architecture diagram, which is mainly composed of two LSTM branches, one of which is used to generate displacement and the other is used to generate rotation matrix and finally determines the new joint coordinates.

**Figure 5:** Spatial temporal diagram of the skeleton sequence. Dots represent joints, black dots represent the same joint in different frames, red edges represent spatial edges, and green edges represent temporal edges.

**Figure 6:** Schematic diagram of the distance vector between keypoints.

**Figure 7:** Comparative experiment of the two models on the NTU-RGB + D datasets.

**Figure 8:** Comparative experiment of the four models on the NTU-RGB + D datasets.

**Table 1:** Results on the NTU-RGB + D datasets.

Methods	X-Sub (%)	X-View (%)
HBRNN-L [9]	64.0	59.1
Part-aware LSTM [26]	70.3	62.9
Trust gate ST-LSTM [27]	77.7	69.2
Two-stream RNN [28]	79.5	71.3
STA-LSTM [29]	81.2	73.4
Ensemble TS-LSTM [30]	81.3	74.6
Visualization CNN [11]	82.6	76.0
VA-LSTM [21]	87.6	79.4
ST-GCN [14]	88.3	81.5
SR-TSL [22]	92.4	84.8
HCN [6]	91.1	86.5
PB-GCN [23]	93.2	87.5
AGC-LSTM [31]	95.0	89.2
**Ours**	**95.3**	**89.5**

**Table 2:** Results on the PKU-MMD datasets.

Methods	X-Sub (%)	X-View (%)
STA-LSTM [29]	44.4	13.1
JCRRNN [32]	32.5	53.3
Skeleton boxes [33]	54.8	94.2
Li et al. [34]	90.4	93.7
HCN [6]	92.6	94.2
**Ours**	**92.7**	**94.4**

## Data Availability

The data used to support the findings of this study are available from the corresponding author upon request.
